# Ignorance Is Not Bliss: A Systematic Review on the Impact of Ignoring UK Medical Students During Clinical Placements

**DOI:** 10.7759/cureus.93644

**Published:** 2025-10-01

**Authors:** Hozafa Ali, Usama Ali

**Affiliations:** 1 Medical Education, Northwick Park Hospital, London, GBR; 2 Geriatric Medicine, Queen Elizabeth The Queen Mother Hospital, Margate, GBR

**Keywords:** clinical placement, medical school, medical school program, medical students, neglect

## Abstract

Introduction: Ignoring medical students on clinical placements is a form of mistreatment that is often overlooked. It is unclear how much research has been done on the topic. We performed the first United Kingdom (UK)-based systematic review on the topic of ignoring medical students. We employed a novel technique that incorporated the use of artificial intelligence (AI) to assist with the review.

Methods: With the assistance of AI, Boolean search terms were generated to search through five databases in July 2025. Studies that described UK medical students being ignored were included in the final analysis. Inductive thematic analysis was performed to identify common themes between the studies. The Critical Appraisal Skills Programme (CASP) checklist for qualitative studies and the Mixed Methods Appraisal Tool (MMAT) for mixed-methods studies were utilized to assess study quality.

Results: Six studies met the criteria to be included in the final analysis. Four common themes were identified when it came to ignoring medical students: exclusion from learning opportunities, emotional and professional invisibility, reporting barriers, and conflicting priorities between medical students and staff. Most of the CASP and MMAT points were met for the included studies, although studies had a small sample size, were often single-center studies, and had a skew toward students in the Midlands.

Discussion: This novel AI-assisted systematic review provided vital information on how and why medical students are ignored in the UK. We propose that a vicious cycle exists when it comes to ignoring medical students. Specifically, students feel ignored, which leads to demotivation, ultimately resulting in disengagement. This leads to staff feeling as though students are uninterested, resulting in further ignoring of medical students. There is limited literature on the prevalence of ignoring medical students, and this is something that needs to be explored in the future.

## Introduction and background

Clinical placements are vital for the professional development of medical students [1]. However, many medical students report mistreatment during placements [2]. This can have an impact on student well-being, with students facing burnout or considering career changes [2,3]. Mistreatment can have many forms. This includes physical, verbal, and sexual abuse [4], public humiliation [5], overt racism [6], and sexism [7]. One form of mistreatment that is often overlooked is learner neglect, which involves ignoring medical students [8].

"Learner neglect" remains poorly defined [9-11]. Kloos et al. describe learner neglect as a lack of inclusion of medical students in the clinical environment [12]. Medical students have described various ways in which they have been ignored [13]. This includes being excluded from clinical discussions or being passive observers rather than active participants in ward rounds, theater, or clinic. It is difficult for students to report mistreatment [14]. Reporting being ignored is no exception [15].

It is unclear how much literature exists on the topic. Current papers on the topic often have small sample sizes and are often single-center studies. Existing literature has also mainly been aimed at medical students outside the United Kingdom (UK) [12]. In the UK, medical school curricula typically last four to six years [16]. At least two to three of these years are spent on clinical placements. Thus, there is the potential for UK medical students to feel ignored for half their time at medical school. This is likely to have emotional, academic, and financial implications.

There is therefore a need to explore the topic of ignoring UK medical students. To the best of our knowledge, there has been no systematic review on the topic. We therefore propose to address this gap within the literature. Specifically, our aims are 1) to identify common themes within the literature when it comes to ignoring UK medical students and 2) to evaluate the quality of current literature on the topic.

## Review

Methods

Overview

We opted to undertake a systematic review on the topic of ignoring medical students in the UK. We endeavored to adhere to the Preferred Reporting Items for Systematic and Meta-Analysis (PRISMA) 2020 guidelines [17]. The review process involved two independent reviewers. Where disagreements occurred, these were discussed and resolved. Artificial Intelligence (AI; ChatGPT-OpenAI o4-mini, OpenAI, Inc., San Francisco, CA) was also used to enhance the review process. The human reviewers oversaw this. The Appendix gives examples of some of the prompts given to AI through the process.

Search Strategies and Electronic Databases

We developed a search string that encompassed four main concepts: 1) medical students, 2) neglect/ignoring/incivility, 3) clinical placements/teaching, and 4) UK setting. We used the Boolean operator "AND" to combine each of these concepts. AI was utilized to help develop synonyms for each concept. This was reviewed by a human and refined. The Boolean operator "OR" was used for the synonyms (Table 1). Using filters, we ensured that the search only included literature from January 2000 to June 2025. We searched electronic databases including Medical Literature Analysis and Retrieval System Online, Embase, Cumulated Index in Nursing and Allied Health Literature, Education Resources Information Center, and PsycINFO.

**Table 1:** Boolean search criteria for each database CINAHL: Cumulated Index in Nursing and Allied Health Literature; ERIC: Education Resources Information Center; MEDLINE: Medical Literature Analysis and Retrieval System Online

Database	Search criteria
MEDLINE	(“Students, Medical"[Mesh] OR medical student*[tiab] OR undergraduate medic*[tiab] OR clinical student*[tiab]) AND ("Neglect (Psychology)"[Mesh] OR "Rudeness"[Mesh] OR neglect*[tiab] OR ignore*[tiab] OR excluded[tiab] OR exclusion[tiab] OR incivilit*[tiab] OR microaggress*[tiab] OR unresponsiv*[tiab] OR "left out"[tiab]) AND ("Clinical Clerkship"[Mesh] OR "Medical Education"[Mesh] OR placement*[tiab] OR clerkship*[tiab] OR "clinical teach*"[tiab] OR "clinical learn*"[tiab] OR ward[tiab] OR hospital[tiab] OR "clinical environment"[tiab]) AND (United Kingdom[tiab] OR UK[tiab] OR England[tiab] OR Scotland[tiab] OR Wales[tiab] OR "Northern Ireland"[tiab]) Filters: Publication date from 2000/01/01 to 2025/07/10; English
Embase	1. 'medical student'/exp OR (medical student* OR undergraduate medic* OR clinical student*).ti,ab. 2. 'neglect'/exp OR 'rudeness'/exp OR (neglect* OR ignore* OR excluded OR exclusion OR incivilit* OR microaggress* OR unresponsiv* OR "left out").ti,ab. 3. 'clinical clerkship'/exp OR 'medical education'/exp OR (placement* OR clerkship* OR "clinical teach*" OR "clinical learn*" OR ward OR hospital OR "clinical environment").ti,ab. 4. (United Kingdom OR UK OR England OR Scotland OR Wales OR "Northern Ireland").ti,ab. 5. 1 AND 2 AND 3 AND 4 Limit to: 2000–2025; English language
CINAHL	(MH "Students, Medical+" OR medical student* OR undergraduate medic* OR clinical student*) AND (MH "Neglect+" OR MH "Rudeness+" OR neglect* OR ignore* OR excluded OR exclusion OR incivilit* OR microaggress* OR unresponsiv* OR "left out") AND (MH "Clinical Clerkship+" OR MH "Medical Education+" OR placement* OR clerkship* OR clinical teach* OR clinical learn* OR ward OR hospital OR "clinical environment") AND (United Kingdom OR UK OR England OR Scotland OR Wales OR "Northern Ireland") Limiters: Publication Date 20000101–20250710; English Language; Peer Reviewed
ERIC	(DE "Medical Students" OR medical student* OR undergraduate medic* OR clinical student*) AND (DE "Incivility" OR neglect* OR ignore* OR excluded OR exclusion OR incivilit* OR microaggress* OR unresponsiv* OR "left out") AND (DE "Clinical Experience" OR DE "Clinical Teaching" OR placement* OR clerkship* OR clinical teach* OR clinical learn* OR ward OR hospital OR "clinical environment") AND (United Kingdom OR UK OR England OR Scotland OR Wales OR "Northern Ireland") Filters: Publication Year 2000–2025; English Language
PsycINFO	1. DE "Students, Medical" OR (medical student* OR undergraduate medic* OR clinical student*).ti,ab. 2. DE "Neglect (Psychology)" OR DE "Rudeness" OR (neglect* OR ignore* OR excluded OR exclusion OR incivilit* OR microaggress* OR unresponsiv*).ti,ab. 3. DE "Clinical Experience" OR DE "Clinical Teaching" OR DE "Medical Education" OR (placement* OR clerkship* OR clinical teach* OR clinical learn* OR ward OR hospital OR "clinical environment").ti,ab. 4. (United Kingdom OR UK OR England OR Scotland OR Wales OR "Northern Ireland").ti,ab. 5. 1 AND 2 AND 3 AND 4 Limits: 2000–2025; English

Study Selection

After applying the search criteria, records were retrieved, and duplicates were removed with the assistance of AI. The two independent reviewers then screened the remaining records using the abstract and title alone. The remaining manuscripts were then retrieved and read in full. The articles were further narrowed down as per the criteria described below. The remaining articles were those that were used in the final review. If disagreements occurred between the reviewers, discussions were held either in person or virtually until a consensus was reached.

We included articles on both undergraduate and graduate-entry medical students within the UK. Articles that had information on the experience of medical students being ignored, excluded, or neglected were included. We excluded articles that primarily investigated students in their preclinical years, non-UK-based medical students, and those with little to no information on the topic of ignoring medical students. We also excluded articles that were not in English, were published before 2000, and for which the full text was not easily available. Review articles and commentaries that did not include student data were also excluded.

Data Synthesis and Quality of Papers

Inductive thematic synthesis [18] was used to identify common themes between the studies. This involved two stages. In the first stage, the human reviewers identified relevant findings within the articles. We prompted the AI model to suggest codes for each finding. The human reviewers reviewed these codes to ensure they were relevant and accurate. The remaining codes were then analyzed and merged to create descriptive themes.

Given the paucity of literature, we did not exclude any study for poor quality. However, the Critical Appraisal Skills Programme (CASP) checklist [19] (for qualitative studies) and the Mixed Methods Appraisal Tool (MMAT; for mixed-method studies) [20] were used to assess study quality.

Results

Study Characteristics and Included Studies

From our search string, 1,500 results were retrieved (Figure 1). Of these results, 107 were duplicates and were subsequently removed. The titles and abstracts were subsequently screened, and an additional 1,350 results were excluded because they did not meet our inclusion criteria. Of the remaining 43 articles, 15 were removed as they investigated non-UK-based medical students, 20 were removed as they did not mention neglecting/ignoring medical students, and two were removed as they were review articles rather than including any new data. This resulted in six studies being included in the final analysis (Table 2).

**Figure 1:** PRISMA diagram showing how studies were selected for the final analysis PRISMA: Preferred Reporting Items for Systematic reviews and Meta-Analyses; CINAHL: Cumulated Index in Nursing and Allied Health Literature; ERIC: Education Resources Information Center; MEDLINE: Medical Literature Analysis and Retrieval System Online

**Table 2:** Titles, characteristics, and findings of the studies that were included in the final analysis

Study	Type of study	Number of participants	Key findings related to ignoring medical students
Webster et al. [21]	Reflective commentary of medical student	1	Described a lack of protected teaching time, teaching being given in an “ultra-rapid” way, and doctors being too busy to acknowledge or teach medical students
Morrison et al. [22]	Qualitative study of focused interviews of medical students	20	Students from minority ethnic backgrounds described reduced acknowledgement from staff, being sidelined from learning opportunities, microaggressions secondary to being excluded, and feeling “invisible” on their clinical placements
Morrison et al. [23]	Qualitative study of focused interviews of medical students	24	Ethnic minority students reported reduced involvement in clinical tasks, limited feedback, and being overlooked for learning opportunities compared to their White peers. This was especially true if clinical teachers were of different ethnic backgrounds
Morrison et al. [24]	Mixed-methods study: survey and focused interview of medical students	362 (survey); 17 (focused group interview)	Several reports from students have been excluded from clinical tasks based on their ethnicity (e.g., by patients), lack of supervision, and teaching time. 59.1% of respondents to a questionnaire reported a lack of confidence in reporting mistreatment
Griffin and Baverstock [25]	Qualitative study: online questionnaire of student experiences	50	12/50 students reported mistreatment by being excluded or dismissed. Students described being ignored as individuals despite trying to integrate into clinical teams. In addition, students were sidelined from clinical opportunities. Students did not report such instances, worrying that being ignored did not constitute a “bad” form of mistreatment
Taylor et al. [26]	Qualitative study: integrative phenomenological analysis	7	Students being ignored by doctors was the “most frequent” barrier faced by students and was often due to a lack of time that doctors had to teach

Thematic Analysis

Inductive thematic analysis revealed four main themes when it came to ignoring medical students: 1) exclusion from learning opportunities, 2) emotional and professional invisibility, 3) reporting barriers, and 4) conflicting priorities.

Exclusion From Learning Opportunities

Across studies, a common theme of being ignored was that of being sidelined from educational opportunities [21-25]. For example, Webster et al. describe occasions where there was little teaching time for medical students, no teacher turning up for scheduled teaching, and a lack of mentorship [21]. Griffin and Baverstock, meanwhile, describe an example of a student being excluded from doing clinical skills [25]. Such instances stemmed from clinical staff assuming the lack of competence of students, thus not allowing them to get involved. The impact of such examples was that students would feel as though they were not part of the team, thus feeling neglected.

Worryingly, Morrison et al.'s studies have provided evidence to suggest that exclusion from learning opportunities may occur due to racial microaggressions [22-24]. Both patients and clinical educators have a role to play in this. In one instance, a British Asian student reported that patients would not be seen by him but would interact with White students [22]. Other students explained that clinical educators of a similar ethnic background would be more willing to provide bedside teaching compared to those of different backgrounds [23]. While there is not much data in the literature commenting on prevalence, Morrison et al.'s mixed-methods study suggests that 89.8% of Black and minority ethnic medical students experienced racial microaggressions [24]. It is not clear how many of these students specifically experienced neglect.

Emotional and Professional Invisibility

In addition to being overlooked for clinical opportunities, students in the studies also described emotional and professional invisibility, which is characterized by not being acknowledged and feeling unseen [21-26]. Examples included being made to sit quietly in clinics without acknowledgement or consultants not taking the time to learn students' names [21]. In Griffin et al.'s paper, students reported that doctors and nurses often completely ignored the presence of medical students. In one case, a student tried to introduce themselves, only for the medical team to not make eye contact with the student and ask them to find another doctor. This was described as "hostile," "rude," "unwelcoming," and "discouraging" for the student. Webster et al. shared similar sentiments and also expressed feelings of discouragement when such emotional and professional invisibility was encountered [21].

More passive forms of emotional invisibility are also evident. Taylor et al. described instances of students striving to participate in clinical discussions [26]. However, despite this, clinical teachers would try to answer questions as quickly as possible, so that they do not have to engage with the student. This made students feel like a "nuisance."

Morrison et al.'s studies once again provide evidence to suggest that ethnic minority medical students may be more prone to experiencing emotional and professional invisibility [22-24]. In both Morrison et al.'s qualitative and mixed-methods studies, there have been examples of ethnic minority medical students not receiving the same amount of attention from their consultants compared to their White counterparts [22,24]. Conversely, there was an example of an Asian medical student who reported feeling less invisible when their consultants were of the same ethnic background [23]. Such consultants were described as being more "paternal" and "nurturing." Similar sentiments were shared by Black medical students [24].

Reporting Barriers

Fifty percent of medical students faced barriers to reporting incivility (including being ignored) in Griffin et al.'s questionnaire [25]. Similarly, Morrison et al.'s mixed-methods study showed that 59.1% of students lacked confidence in reporting such instances [24]. Various reasons were attributed to this.

There was some evidence of students not wanting to report being ignored, as it did not seem as "bad" as other forms of mistreatment [25]. There was, therefore, a fear that medical schools would not take such complaints seriously. This fear was more pronounced in those students from ethnic minority backgrounds [22]. In these cases, students shared examples of how they were perceived to be too "sensitive" when reporting such instances.

Some students were fearful that they would get into trouble if they were to report [25]. In these cases, students alluded to feeling as though they were at the bottom of the hierarchy of clinical staff. Subsequently, students felt as though they were not part of the team, making it harder to report [25,26].

The overall negative experiences of medical students in reporting incivility led to students having a lack of trust in their institutions [22]. This appears to lead to a snowballing effect, where students describe feeling worn down and, as a result, no longer having the motivation to report [25].

Conflicting Priorities

A common theme through the studies was the difficulties experienced by clinical staff in balancing service pressures and teaching medical students [21,25,26]. Webster et al., for instance, cited examples of doctors barely having time to sit down, thus making it hard for them to abandon their jobs and teach. In one case, a doctor was given the task of teaching after their fourth night shift, meaning they could not dedicate an appropriate amount of time to teaching.

There were also instances of medical students being told they would "slow the doctors" down [25]. Interestingly, such sentiments would often come from more senior doctors, as evidenced by both Griffin and Baverstock [25] and Taylor et al. [26]. This was even if the junior doctors themselves would try to include medical students [25]. Students themselves also described feeling as though they were a hindrance to doctors, noting how busy the medical team was and how they felt guilty "using up" their time [26].

Quality of Papers

Of the papers included in the final analysis, four of six (66.7%) were qualitative studies, one (16.6%) was a mixed-methods study, and one (16.6%) was a personal reflective commentary. We decided to include the reflective commentary in the final analysis as it captured the voice of medical students in a similar way to the qualitative studies.

We used the CASP tool for qualitative studies and the MMAT for the mixed-method study to appraise quality. All the papers had clear research aims, although none of them (apart from the reflective commentary) exclusively looked at the topic of ignoring medical students. This highlights the paucity of literature on the topic within the UK. The methods of collecting data through focused interviews were clearly explained in all the papers, as was explaining how the data were subsequently processed. Reflexivity was at least partially clear in all the qualitative and mixed-method studies, with interviewers being aware of how their biases might influence the results.

A major weakness of the studies was the small sample size of participants. This varied from 1 (in the reflective commentary) to 50 participants in the focused interviews. In addition, all but one paper, Morrison et al. [22], were single-center studies. There was also a geographical skew of the studies, such that the results are more skewed towards students in the Midlands. Table 3 summarizes the quality of the studies.

**Table 3:** Summary of the strengths and weaknesses of the included studies N/A: not available; CASP: Critical Appraisal Skills Program; MMAT: Mixed Methods Appraisal Tool CASP was used for qualitative studies, and MMAT was used for the mixed-methods study

Study	Quality assessment tool	Strengths	Weakness
Webster et al. [21]	N/A: commentary	Clear, personal account of experiences of being neglected. Directly addresses the main question of this review	Experience of only one medical student; written commentary rather than original research, so may not be generalizable
Morrison et al. [22]	CASP	Met 9/10 of the CASP criteria: clear aims; appropriately selected qualitative study design; appropriate research design; adequate data collection; researcher reflexivity considered; ethical issues considered; data analyzed rigorously; clear statement of results; clear value of the paper	1/10 CASP criteria was partially met: recruitment strategy was clearly described. However, recruitment was skewed toward one area of the UK, and it is not clear what area this was
Morrison et al. [23]	CASP	Met 8/10 of the CASP criteria: clear aims; appropriately selected qualitative study design; appropriate research design; adequate data collection; ethical issues considered; data analyzed rigorously; clear statement of findings; clear value of the paper	2/10 CASP criteria partially met: while the study design was appropriate, it was only single-center; reflexivity was evident in that the background of the interviewer was described, but could have been in a bit more detail
Morrison et al. [24]	MMAT	Met 3/5 of the MMAT criteria: adequate rationale for using mixed-methods design; different components of the study adequately answer the research question; the outputs of both qualitative and quantitative aspects of the study are properly interpreted	Partially met 2/5 of the MMAT criteria: unclear if divergences between qualitative and quantitative data were present and addressed; the qualitative part of the study was well described. The quantitative part was also done well, although the survey used did not have any previous psychometric validation. However, this was acknowledged by the authors
Griffin and Baverstock [25]	CASP	Met 7/10 of the CASP criteria: clear aims; appropriate research design; appropriately selected qualitative study design; adequate data collection; ethical issues considered; clear statement of findings; clear value of the paper	3/10 CASP criteria partially met: the recruitment strategy was well described, but there was a lack of validation of responses; reflexivity was only briefly mentioned/acknowledged; while the analysis was, in general, rigorous, the study was hampered by a small sample size and being single-center. However, this was acknowledged by the authors
Taylor et al. [26]	CASP	Met 9/10 of the CASP criteria: clear aims; appropriately selected qualitative study design; research design appropriate; adequate data collection; reflexivity clearly accounted for and very well explained; ethical issues considered; data analyzed rigorously; clear statement of the findings; clear value of the paper	1/10 CASP criteria partially met: while the recruitment strategy was well described, only a small number of students were recruited. This is a harsh analysis, however: the study was a well-designed interpretive phenomenological analysis where small sample sizes are key. Unfortunately, for the sake of the CASP criteria, it must be mentioned and labeled as partially meeting the criteria

Discussion

Ignoring Medical Students

This is the first UK-based systematic review exploring the topic of ignoring medical students. We identified four main themes: exclusion from learning opportunities, emotional/professional invisibility, barriers to reporting such mistreatment, and conflicting priorities of students and educators. These themes interlink with one another.

Medical students can be ignored intentionally or unintentionally, a sentiment shared by Buery-Joyner et al. [8]. The true extent of ignoring medical students is unclear and remains unclear after this review. This is something that should be investigated quantitatively in the future. However, it is clear that service pressures often play a role in either intentional or unintentional ignoring of medical students. Given that service demands are increasing without a proportionate increase in clinical staff [27], the extent of ignoring medical students is likely to increase.

Interestingly, our review highlighted that junior doctors were often less likely to ignore medical students despite service pressures. Indeed, evidence suggests that medical students often find junior doctors to be more approachable on clinical placements compared to senior doctors [28,29]. Perhaps this is because junior doctors remember more clearly the challenges of being a medical student. In some cases, junior doctors were told by their senior colleagues to deprioritize teaching medical students in favor of service demands [25,26]. A supportive environment is key in encouraging junior doctors to act as teachers [30]. Thus, discouraging teaching in this way is likely to have detrimental effects on both medical students and on the teachers who are most willing to teach them.

Although burnout among medical students is well-documented in the literature [31-38], little attention has been paid to the impact of ignoring medical students. As per Maslow’s Hierarchy, "Belonging" is one of the basic needs [39]. By ignoring medical students, this basic need is neglected. It is therefore likely that ignoring medical students has detrimental effects on their mental health. Such detriments may lead to further demotivation of medical students, making them less likely to engage in teaching [40-44]. Clinical teachers may incorrectly perceive such students to be disinterested [45,46]. We propose that this can lead to a vicious cycle: students feel ignored, subsequently become demotivated, which in turn leads to disengagement. This, in turn, leads staff to believe that students are uninterested, resulting in further ignoring of students (Figure 2).

**Figure 2:** Proposed cycle of ignorance Students being ignored leads to them being demotivated, which leads to them becoming disengaged. This leads to staff perceiving students as uninterested, and subsequently, to further ignoring of students Source: This is an original diagram designed and produced by the author Hozafa Ali

Our review yielded similar findings to those in the international literature. Kloos et al. carried out a related systematic review of students in the US [12]. Like the UK, it appears that conflicting priorities contribute to the neglect of medical students in the US. Meanwhile, Valestrand et al. found evidence of professional/emotional invisibility among medical students in Norway [47]. Several other studies worldwide have also shown similar barriers to reporting mistreatment as experienced by UK medical students [14,48-52]. Overall, there are similar themes across the world when it comes to ignoring medical students.

Strengths, Limitations, and the Use of AI

This is the first systematic review on the topic of ignoring medical students in the UK. We believe we had clear aims in exploring this topic and were able to meet these objectives through the review. Namely, this review has helped raise the importance of the topic, identifying important themes to consider. We also strived to follow the PRISMA guidelines when performing this review and appraise the quality of the included papers.

Nevertheless, this review has limitations. Firstly, only six papers were included. However, we do not think that this was due to strict inclusion criteria. Rather, the small number of papers highlights the need for more original research to be done on the topic. Second, very few of the included papers concentrated exclusively on ignoring medical students. Nevertheless, we still had enough information from the papers to include them in the final review. Third, we were unable to find any empirical data on the extent of the problem of ignoring medical students. Finally, of the included papers, there was a geographical skew toward students in the Midlands. This means that the findings of this review may not apply to all students in the UK. Further studies are therefore needed in other parts of the UK.

An increasing amount of attention is being given to the use of AI in systematic reviews [53-56]. Using AI helped save time by defining the search criteria, removing duplicate studies, and facilitating coding to carry out the thematic analysis. When correct prompts were used, this was done accurately.

However, it was important to ensure that a human reviewed every AI step. There was one instance where AI "invented" fake papers when helping to perform the search, and these were only identified after the human reviewers went through the papers manually. This highlighted the importance of giving clear prompts to the AI tool. In this case, it was important to highlight that the search we wanted to perform was not for illustrative purposes only. Once this was clarified, the AI tool worked appropriately. This is something future researchers should consider when using AI to assist in systematic reviews.

The AI model used should also be considered. Models such as Elicit (Elicit, San Francisco, CA) [55], for example, have been designed specifically to assist with systematic reviews, and therefore, it is a model we will consider in the future. We opted to use OpenAI o4-mini (ChatGPT) as it is the most popular AI model in use [57], and we were keen to explore its functionality in assisting with a systematic review. It is unclear which model is best to use. Helms Andersen et al. recently showed comparable outcomes in performance of both Elicit and ChatGPT [58]. Data on the topic is limited, however, and it will be exciting to see how AI influences systematic reviews in the future.

## Conclusions

This systematic review highlighted some key issues when it comes to ignoring medical students in the UK. Ignoring medical students can include things like overlooking them for clinical teaching. Unfortunately, it can also encompass ignoring them as human beings, making them feel invisible. A lot of this stems from the fact that UK doctors do not have enough time to teach or, in some cases, even acknowledge medical students. Although this clearly has a negative impact on medical students, several remain scared to report it, highlighting fears of repercussion as people may not perceive it to be "serious" enough. Further work is required to highlight the extent of the problem.

## Appendices

**Table 4:** Examples of prompts given to the AI model Please note that the list of prompts is not exhaustive AI: artificial intelligence

Method step	AI prompt example (list not exhaustive)	Human validation steps involved
Developing search term	Please generate 30 synonyms for the concept “medical student.” The synonyms are for potential use in a search of an online database for a systematic review on the topic of ignoring medical students	Manually reviewing the suggested synonyms, removing irrelevant synonyms, and then selecting the final ones to be included in the final search
Developing search term	Please do the same for the concept of “neglect/incivility/ignoring”	Manually reviewing the suggested synonyms, removing irrelevant synonyms, and then selecting the final ones to be included in the final search
Developing search term	Please again do the same for the concept of “Clinical placements/teaching”	Manually reviewing the suggested synonyms, removing irrelevant synonyms, and then selecting the final ones to be included in the final search
Inductive thematic analysis	An excerpt from the article above [uploaded] is as follows: [excerpt copied and pasted]. Please generate 1-3 code words for the extract that can be used for the systematic review such that inductive thematic analysis can be performed. Please try to keep the codes between 1-3 words	Code words were reviewed, merged if necessary, and removed if irrelevant
Inductive thematic analysis	In response to AI asking if we would like the AI model to search for excerpts itself: "Yes, please help with other excerpts as well and we can compare your excerpts with the ones we had in mind"	Code words were reviewed, merged if necessary, and removed if irrelevant. AI-extracted excerpts were compared to our excerpts to confirm they were relevant to the review
